The article "Diabetes and Overexpression of proNGF Cause Retinal Neurodegeneration via Activation of RhoA Pathway" was retracted in 2017. Reasons: an official misconduct investigation; misconduct by an author; duplicated images.

# Diabetes and Overexpression of proNGF Cause Retinal Neurodegeneration via Activation of RhoA Pathway

**DOI:** 10.1371/journal.pone.0054692

**Published:** 2013-01-24

**Authors:** Mohammed M. H. Al-Gayyar, Barbara A. Mysona, Suraporn Matragoon, Mohammed A. Abdelsaid, Mona F. El-Azab, Ahmed Y. Shanab, Yonju Ha, Sylvia B. Smith, Kathryn E. Bollinger, Azza B. El-Remessy

**Affiliations:** 1 Program in Clinical and Experimental Therapeutics. College of Pharmacy, University of Georgia, Athens, Georgia, United States of America; 2 Department of Pharmacology and Toxicology, Georgia Health Sciences University, Augusta, Georgia, United States of America; 3 Department of Cell Biology and Anatomy, Georgia Health Sciences University, Augusta, Georgia, United States of America; 4 Department of Ophthalmology, Georgia Health Sciences University, Augusta, Georgia, United States of America; 5 Vision Discovery Institute, Georgia Health Sciences University, Augusta, Georgia, United States of America; 6 Charlie Norwood Veterans Affairs Medical Center, Augusta, Georgia; Universidade Federal do Rio de Janeiro, Brazil

## Abstract

Our previous studies showed positive correlation between accumulation of proNGF, activation of RhoA and neuronal death in diabetic models. Here, we examined the neuroprotective effects of selective inhibition of RhoA kinase in the diabetic rat retina and in a model that stably overexpressed the cleavage-resistance proNGF plasmid in the retina. Male Sprague-Dawley rats were rendered diabetic using streptozotosin or stably express cleavage-resistant proNGF plasmid. The neuroprotective effects of the intravitreal injection of RhoA kinase inhibitor Y27632 were examined *in vivo*. Effects of proNGF were examined in freshly isolated primary retinal ganglion cell (RGC) cultures and RGC-5 cell line. Retinal neurodegeneration was assessed by counting TUNEL-positive and Brn-3a positive retinal ganglion cells. Expression of proNGF, p75^NTR^, cleaved-PARP, caspase-3 and p38MAPK/JNK were examined by Western-blot. Activation of RhoA was assessed by pull-down assay and G-LISA. Diabetes and overexpression of proNGF resulted in retinal neurodegeneration as indicated by 9- and 6-fold increase in TUNEL-positive cells, respectively. *In vitro*, proNGF induced 5-fold cell death in RGC-5 cell line, and it induced >10-fold cell death in primary RGC cultures. These effects were associated with significant upregulation of p75^NTR^ and activation of RhoA. While proNGF induced TNF-α expression *in vivo*, it selectively activated RhoA in primary RGC cultures and RGC-5 cell line. Inhibiting RhoA kinase with Y27632 significantly reduced diabetes- and proNGF-induced activation of proapoptotic p38MAPK/JNK, expression of cleaved-PARP and caspase-3 and prevented retinal neurodegeneration *in vivo* and *in vitro*. Taken together, these results provide compelling evidence for a causal role of proNGF in diabetes-induced retinal neurodegeneration through enhancing p75^NTR^ expression and direct activation of RhoA and p38MAPK/JNK apoptotic pathways.

The article "Diabetes and Overexpression of proNGF Cause Retinal Neurodegeneration via Activation of RhoA Pathway" was retracted in 2017. Reasons: an official misconduct investigation; misconduct by an author; duplicated images.

## Introduction

Our recent studies showed significant accumulation of proNGF that was positively correlated with accelerated retinal neurodegeneration in models of diabetes [1], [2]. Our studies demonstrated a mechanism by which diabetes-induced peroxynitrite impairs the activity and expression of MMP-7, an extracellular enzyme involved in maturation of NGF leading to accumulation of the proNGF [2]. While mature NGF mediates neuronal cell survival through binding TrkA and p75^NTR^ receptors, proNGF can promote neuronal apoptosis because of its high affinity to p75^NTR^ [3], [4]. It has been shown that the outcome of the neurotrophin signaling, neurotrophic or apoptotic can be dependent upon relative levels of its receptors [5], [6]. Our studies in diabetic human and rat retina demonstrated tyrosine nitration and inhibition of the survival receptor TrkA and upregulation of the proapoptotic receptor p75^NTR^ [1], [7].

In non-diabetic models, overexpression of p75^NTR^ has been shown to constitutively activate RhoA leading to neuronal death via activation of p38MAPK pathway [8]–[12]. Rho family GTPases are monomeric G-proteins that act as key transducers of integrin signaling [13] and growth factor signaling [2], [14], [15]. RhoA is a major small GTP-binding protein that acts as a molecular switch to play either a pro-death or pro-survival role in the nervous system depending on both the type of neuron and the particular neurodegenerative insult involved (for review [16]). Prior report showed that activation of RhoA can directly induce neuronal death in excitotoxic model [9]. Yet, whether RhoA activation can induce retinal neurodegeneration in response to proNGF or diabetic insult remains unexplored.

The MAPK family includes four groups: extracellular signal regulated kinase (ERK), c-Jun N-terminal kinase/stress-activated protein kinase (JNK/SAPK), p38 and ERK5. MAPKs are activated in response to a wide range of extracellular stimuli including growth factors, serum, hormones, cytokines and others more related to stress responses (i.e. UV radiation, X-rays, heat and osmotic shock), and they are involved in many different cellular processes such as embryogenesis, proliferation, differentiation, transformation and apoptosis (for review [17]). In particular, JNK/SAPK and p38 MAPK pathways have been shown to play an important role in neuronal apoptosis in various models including neurotoxicity, diabetes, neurotrophic deprivation or excessive proNGF *in vitro* [1], [18]–[21] and *in vivo* [2], [7], [22].

The article "Diabetes and Overexpression of proNGF Cause Retinal Neurodegeneration via Activation of RhoA Pathway" was retracted in 2017. Reasons: an official misconduct investigation; misconduct by an author; duplicated images.

In this study, we aimed to elucidate molecular events by which proNGF contributes to diabetes-induced retinal neurodegeneration. In particular, we examined the specific role of RhoA kinase activation as downstream signaling pathway in response to proNGF. Here, we demonstrate the first evidence of the neuroprotective effects of inhibiting RhoA kinase in models of diabetes as well as overexpression of proNGF in healthy rat retina and cultures of primary retinal ganglion cells.

## Materials and Methods

### Animal preparation

All procedures with animals were performed in accordance with the ARVO Statement for the Use of Animals in Ophthalmic and Vision Research, and the Charlie Norwood VA Medical Center Animal Care and Use Committee. Three sets, a total of 60 Male Sprague-Dawley rats (∼250 g body weight) from Harlan laboratories (Indianapolis, IN) were housed in a 12 h light/dark cycle at a controlled temperature and humidity with free access to food and water.

### Induction of diabetes in rats

Rats (24) were randomly assigned to control, treated control, diabetic or treated diabetic groups. Diabetes was induced by intravenous injection of streptozotocin (60 mg/kg). Detection of glucose in urine and blood glucose levels >13.9 mmol/l indicated diabetes. Treatment was initiated 2-weeks after confirmation of diabetic status and continued for additional 3 weeks for various endpoints. Treated control and diabetic rats were injected intravitreally with the specific RhoA kinase inhibitor Y27632 (100 nmole/eye) once/week. Treatment with Y27632 did not alter body weight in control (360±4 vs 370±22) or diabetic animals (295±20 vs 286±14). Treatment with Y27632 did not alter blood glucose levels in control (120±8 vs 125±10) or diabetic animals (421±20 vs 418±22).

### ProNGF overexpression studies

Rats (36) were randomly assigned to receive intravitreal injection with pGFP plasmid (5 µg/eye), pGFP-proNGF123 construct (5 µg/eye) or combination of pGFP-proNGF123 plasmid and the specific RhoA kinase inhibitor Y27632 (100 nmole/eye) from Cayman (Ann Arbor, MI). Electroporation was performed as described previously by our group [23]. Rats were sacrificed after 1-week and eyes were enucleated and processed for further analyses.

### Tissue culture studies

#### Primary retinal ganglion (RGC) cells

RGC were isolated from retinas of 2-day-old mice by immunopanning techniques as previously described by our group [24]. Cells were maintained in culture for 2 days in neurobasal medium containing 50 µg/ml BDNF, 10 µg/ml CNTF, 10 µg/ml Forskolin and 10 µg/ml bFGF, in the 30 mm dishes coated with poly D-lysine and laminin. RGC were rinsed with neurobasal medium without growth factors and equilibrated in the same medium for treatment. RGC were treated with mouse mutant proNGF (50 ng/ml) from Alomon (Israel) in the presence of Y27632 (1 µM) for overnight. For G-LISA studies, cells were harvested after 6-hours.

The article "Diabetes and Overexpression of proNGF Cause Retinal Neurodegeneration via Activation of RhoA Pathway" was retracted in 2017. Reasons: an official misconduct investigation; misconduct by an author; duplicated images.

#### Adult mouse retinal mixed neuronal culture

Adult mouse retinal mixed neuronal culture was prepared as previously described [25]. 20 retinas from 6week-old mice were dissected in Hank's buffered-saline solution (HBSS) and incubated at 37°C for 10 min in a digestion solution containing papain (10 U/mL; Worthington, Lakewood, NJ) and L-cysteine (0.3 mg/mL; Sigma) in HBSS. Retinas were rinsed and triturated in HBSS containing bovine serum albumin (1 mg/mL; Sigma) and DNase (0.2 mg/mL; Sigma). Dissociated cells were passed through a strainer (40-µm nylon net; Falcon, Bedford, MA) and collected by centrifugation. Cells were resuspended in a 1 mL neurobasal medium (Invitrogen) with B27 supplement (Invitrogen). Cells were seeded into slide chamber and used characterized p75^NTR^ expression in RGC cells using immunolocalization techniques.

#### Retinal ganglion cell line (RGC-5)

Retinal ganglion cell line (RGC-5), was a kind gift from Dr. N. Agarwal (Department of Cell Biology UT Health Science Center, Fort Worth, TX) and have been previously characterized [26]. Cells were grown to confluence in complete medium (DMEM with 6% FBS and 10% penicillin/streptomycin) then switched to serum free media. Cells were treated with mouse mutant proNGF (50 ng/ml) from Alomon (Israel) in the presence or absence of Y27632 (1 µM) for overnight.

### Immunolocalization studies

OCT-frozen sections (10 µm) of eyes were fixed using 2%PFA in PBS and reacted with polyclonal p75^NTR^ (Millipore, Billerica, MA), monoclonal anti-Brn-3a antibody (specific RGC marker, Santa Cruz) or monoclonal anti-Thy-1, a neuronal marker, antibody (Santa Cruz) overnight followed by Texas-red or Oregon-green-conjugated goat anti-mouse or goat anti-rabbit antibodies (Invitrogen, Carlsbad, CA). Images (n = 4–6 in each group) were collected using AxioObserver.Z1 and confocal Microscope (Zeiss, Germany).

### Evaluation of retinal cell death in vivo

TUNEL assay was performed to detect retinal cell death by using immunoperoxidase staining (ApopTag-Peroxidase), in whole-mount retina as described previously by our group [2], [7]. Briefly, formalin-fixed retinas were flat-mounted, dehydrated in ethanol, defatted by xylenes and rehydrated. After permeabilization, TUNEL-HRP staining with 3-amino-9-ethylcarbazole was performed following the manufacturer's instructions.

The article "Diabetes and Overexpression of proNGF Cause Retinal Neurodegeneration via Activation of RhoA Pathway" was retracted in 2017. Reasons: an official misconduct investigation; misconduct by an author; duplicated images.

### Determination of RGC death in vitro

TUNEL-positive cells were determined using TUNEL fluorescence (ApopTag-Fluorescein) and counterstained with DAPI (blue) or Propidium Iodide (red). The total number of TUNEL-positive cells was counted and expressed as percentage of TUNEL positive cells/total number of cells in various groups.

### Counting number of total retinal neuronal and ganglion cells

Total cells in ganglion cell layer (GCL) was counted as described previously by our group [27]. Briefly, OCT frozen retinal sections were stained with Hematoxylin and Eosin (H/E) for light microscopy. The nuclei in the GCL, not including nuclei in the vessels, were counted in four locations in the retina including both sides of the optic nerve (posterior) and mid-retina (central) in a masked manner. Since neuronal cells in GCL contain RGC and amacrine cells, ganglion cells were labeled using Brn3a monoclonal antibody (Santa Cruez) and total number of cells were counted using DAPI. Cells in the GCL were counted from ora serrata to ora serrate (retina length). RGCs were identified as cells positive for Brn3a, a specific RGC marker and DAPI positive in the GCL. Number of RGC was normalized to retina length (mm) in each section. For each animal two sections were counted, one near the optic nerve and one located more peripherally. Four to six animals from each group and two fields for each location were used. Retinas were imaged by AxioObserver.Z1 Microscope (Zeiss, Germany).

### Retinal protein extraction and Western blot (WB) analysis

Retinas were isolated and homogenized in RIPA buffer as described previously [7]. Samples (50 µg protein) were separated by SDS-PAGE and electroblotted to nitrocellulose membrane. Antibodies for p75^NTR^ (Millipore, Billerica, MA), JNK, p-JNK (Santa Cruz Biotechnology, Santa Cruz, CA), p-p38, p38, cleaved caspase-3 (Cell Signaling, Danvers, MA) and cleaved PARP (BD Bioscience Pharmingen, San Diego, CA) were used. Membranes were reprobed with β-actin (Sigma-Aldrich, St. Louis, MO) to confirm equal loading. The primary antibody was detected using a horseradish peroxidase-conjugated sheep anti-rabbit antibody (GE Healthcare, Piscataway, NJ) and enhanced chemiluminescence. The films were scanned and the band intensity was quantified using densitometry software (alphEaseFC) and expressed as relative optical density (ROD).

### Quantitative real time PCR

Retinal mRNA was prepared according to the manufacturer's instructions as described in our previous study [7]. The One-Step qRT-PCR Invitrogen kit was used to amplify 10 ng retinal mRNA from each sample. PCR primers were designed to amplify TNF-α: 5′GGGTGATCGGTCCCAACA′ and reverse primer 5′TGGGCTACGGGCTTGTCA. Primers were designed to amplify p75^NTR^: 5′-GCA GCT CCC AGC CTG TAG TG-3′ and reverse primer 5′-TAG GCC ACA AGG CCC ACA AC-3′. Amplification of 18S rRNA was used as an internal control. Quantitative PCR was performed using a Realplex Master cycler (Eppendorf, Germany). TNF-α expression was normalized to the 18S level in each sample and expressed as relative expression to control.

The article "Diabetes and Overexpression of proNGF Cause Retinal Neurodegeneration via Activation of RhoA Pathway" was retracted in 2017. Reasons: an official misconduct investigation; misconduct by an author; duplicated images.

### Retinal RhoA kinase activity

GTPase activity was assessed by pull down assay. As previously described, retinas or retinal ganglion cells were homogenized in assay buffer [28]. Homogenates were incubated with agarose conjugated rhotekin-RBD (Millipore, Billerica, MA,) for 45 min at 4°C and washed three times with lysis buffer. Agarose beads were boiled in Laemmli reducing sample buffer to release active RhoA. Bound RhoA was detected by Western blot using anti-RhoA monoclonal antibody (Millipore, Billerica, MA).

### G-LISA detection of RhoA GTPase activity in primary RGC cultures

G-LISA detection of RhoA GTPase activity in primary RGC cultures was performed using a G-LISA kit from (Cytoskeleton, Denver, CO) according to manufacture protocol. RGC cells were washed with PBS, resuspended in lysis buffer from the kit and harvested from the dishes with cell scraper. Total protein concentration in each lysate was determined by protein assay reagent from the kit. The G-LISA's contains a RhoA-GTP-binding protein immobilized on microplates. Bound active RhoA was detected with a specific antibody and luminescence, which was quantified using a microplate reader (BioTek Instruments) after removing the reaction mixture.

### Data analysis

The results were expressed as mean ± SEM. Differences among experimental groups were evaluated by ANOVA followed by Tukey-Kramer Multiple comparison test. Significance was defined as P<0.05.

## Results

### Inhibiting RhoA blocked diabetes- and proNGF-induced neuronal death *in vivo*

Our previous studies in STZ-diabetic model showed accumulation of proNGF and neuronal cell death that were positively correlated with activation of RhoA [1], [2]. Here we tested the direct neuroprotective effects of inhibiting Rho kinase in response to diabetes (5-weeks) or proNGF overexpression (1-week). As shown in Figure 1A, diabetic rat flat-mounted retina showed ∼9-fold increase in the TUNEL-HRP-positive cells counted in each retina as compared with non-diabetic controls (Fig. 1A, 1B). Intravitreal treatment with the RhoA kinase inhibitor Y26732 blocked apoptotic effects of diabetes in the rat retina. To dissect the role of proNGF in retinal neurodegeneration apart from the complex diabetic milieu, overexpression of the cleavage-resistant proNGF construct was used as described previously [23]. As shown in Figure 1C, overexpression of proNGF caused ∼6-fold increase in TUNEL-positive cells compared to the GFP-control. Overexpression of proNGF also caused 20 and 30% reduction of total neuronal cells in ganglion cell layer (GCL) in both central and posterior retina, respectively (Fig. 2A, 2C). Since GCL contains a mixed population of retinal ganglion cells and displaced amacrine cells, RGCs were labeled and counted using Brn3a antibody (Fig. 2B) and normalized to retina length. As shown in Figure 2D, overexpression of proNGF caused significant reduction (60%) of RGC count compared to pGFP controls. Co-treatment with the RhoA kinase inhibitor Y26732 blocked proNGF effects and protected retinal ganglion cells from cell death.

The article "Diabetes and Overexpression of proNGF Cause Retinal Neurodegeneration via Activation of RhoA Pathway" was retracted in 2017. Reasons: an official misconduct investigation; misconduct by an author; duplicated images.

**Figure 1:** Inhibiting Rho kinase blocked proNGF and diabetes-induced retinal neurodegeneration. **A,B.** Representative images and statistical analysis of TUNEL-HRP-positive cells counted in each retina flat-mount showing ∼9-fold increased number of cell death in retinas from 5 weeks diabetic rats as compared with the controls (n = 4–5). **C.** Statistical analysis of total number of TUNEL-HRP-positive cells counted in each retina showing ∼6-fold increase of cell death in retinas that overexpress proNGF as compared with the GFP controls (n = 4–5). Treatment with the selective Rho kinase inhibitor Y27632 blocked these effects in diabetic and proNGF overexpression and did not affect the control groups. * = significant difference as compared with the rest of the groups at p<0.05. C, control; D, diabetic; Y, Y27632.

**Figure 2:** Inhibiting Rho kinase blocked proNGF-induced neuronal cell death. **A,C.** Representative images and statistical analysis of rat retina sections stained with H/E showing a reduction in total number of neuronal cells in the GCL in rats injected with proNGF as compared with pGFP-controls in central and posterior retina (n = 4, 200× magnification). **B,D.** Representative images and statistical analysis of rat retina sections stained with anti-Brn3, specific RGC marker, showing a reduction in number of RGC in proNGF as compared with GFP-controls in central and posterior retina (n = 6, 400× magnification). Treatment with Y27632 blocked these effects in proNGF injected rats. * = significant difference as compared with the rest of the groups at p<0.05. GCL, ganglion cell layer; IPL, inner plexiform layer; INL, inner nuclear layer; ONL, outer nuclear layer.

### Inhibiting RhoA blocked proNGF-induced death in primary RGC cultures

We next investigated the neuroprotective effects of Y27632 in RGC cultures. We compared the apoptotic effects of proNGF on freshly isolated primary RGC to the cell line RGC-5. Our studies in RGC-5 showed ∼5-fold increase in the number of TUNEL-positive cells in response to mutant proNGF (50 ng/ml) compared to controls (Fig. 3A, 3B). Studies using primary RGC cells showed higher sensitivity (>10-fold) to apoptotic effects of proNGF (Fig. 3C, 3D) compared to controls. Co-treatment with Y27632 (1 µM) protected RGC in proNGF-treated group but had no effect on control cells.

The article "Diabetes and Overexpression of proNGF Cause Retinal Neurodegeneration via Activation of RhoA Pathway" was retracted in 2017. Reasons: an official misconduct investigation; misconduct by an author; duplicated images.

**Figure 3:** Inhibiting RhoA blocked proNGF-induced death in primary RGC cultures. **A,B.** Representative images and statistical analysis showing ∼5-fold increase in TUNEL-positive cells in RGC-5 cells in response to mutant proNGF (50 ng/ml) (200× magnification). **C,D.** Representative images and statistical analysis showing ∼10-fold increase in TUNEL-positive cells in primary RGC cultures in response to mutant proNGF (50 ng/ml) (200× magnification). Co-treatment with Y27632 (1 µM) protected RGC in proNGF-treated group but had no effect on control cells. * = significant difference as compared with the rest of the groups at p<0.05 (n = 4). C, control; Y, Y27632.

### Diabetes and overexpression of proNGF induced expression of p75^NTR^ in vivo and in vitro

Our previous analyses showed that diabetes and proNGF overexpression induce p75^NTR^ expression [1], [2], [7], [23]. We examined the effects of inhibiting Rho kinase on p75^NTR^ expression. As shown in Figure 4A–B, diabetes caused 2-fold and proNGF caused 1.5-fold increase in p75^NTR^ expression compared to controls. These effects were partially but significantly reduced by treatment with Y27632. In addition, prominent immunolocalization of p75^NTR^ was observed in GCL and inner retinal layers in proNGF group as compared with pGFP-controls (Fig. 4C). Colocalization of p75^NTR^ with both Brn-3a, specific RGC marker, and Thy-1, neuronal marker, in the ganglion cell layer (Fig. 4D) confirmed the upregulation of p75NTR within retinal ganglion cells. *In vitro*, in comparison to controls, proNGF induced 1.6-fold increase in p75^NTR^ expression in RGC-5 cell line (Fig. 4E) as well as 2.5-fold increase in p75^NTR^ mRNA expression in freshly isolated primary RGC (Fig. 4F). Treatment with Y27632 significantly reduced p75^NTR^ expression in RGC-5. To further confirm p75^NTR^ expression in adult RGC cultures, we isolated mixed neuronal cultures and immunolocalized p75^NTR^ (red) with the specific RGC marker Brn3a (green). As shown in Figure 4G, numerous co-localized RGC cells (yellow) that express p75^NTR^ were detected in the field.

**Figure 4:** Diabetes and overexpression of proNGF induced expression of p75^NTR^ in vivo and in vitro. **A.** WB analysis showing 1.9-fold increase in the expression of p75^NTR^ in diabetic rats as compared with the controls (n = 4–6). **B.** WB analysis of rat retinal lysate showed significant increase in p75^NTR^ expression in rats electroporated with proNGF as compared with those electroporated with GFP (n = 4). **C.** Representative images of rat retina sections showing prominent immunolocalization of p75^NTR^ in GCL and INL in proNGF overexpressing retinas as compared with GFP-controls (400× magnification). **D.** Representative images of rat retina sections showing colocalization between p75^NTR^ in the ganglion cell layer (green) and the specific neuronal marker Thy-1 (red) in the upper pannel or with the specific RGC marker Brn-3a (red)in the lower pannel (400× magnification). **E.** Western blot analysis shwoing 1.6-fold increase in the expression of p75^NTR^ in RGC-5 cells treated with proNGF as compared with the controls (n = 4). **F.** Real-time PCR analysis showing that proNGF induced p75^NTR^ mRNA expression in freshly isolated primary RGC as compared with the control group. Samples of primary RGC cultures were pooled from 4-different cultures. Treatment with Y27632 significantly reduced p75^NTR^ expression *in vivo* and *in vitro*. G. Representative images showing colocalization (yellow arrow heads) of RGC that expressed p75^NTR^ (red) and the specific RGC marker Brn3a (green) in isolated mixed neuronal cultures from adult mice. * = significant difference as compared with the rest of the groups at p<0.05. C, control; GCL, ganglion cell layer; IPL, inner plexiform layer; INL, inner nuclear layer; ONL, outer nuclear layer. C, control.

The article "Diabetes and Overexpression of proNGF Cause Retinal Neurodegeneration via Activation of RhoA Pathway" was retracted in 2017. Reasons: an official misconduct investigation; misconduct by an author; duplicated images.

### ProNGF selectively causes RhoA kinase activation *in vivo* and in RGC cultures

Our studies in the diabetic retina showed positive association between increased proNGF and activation of RhoA [7]. Indeed, diabetic rat retina showed significant increase (2.3-fold) in active RhoA compared to controls (Fig. 5A). Next, we examined the effect of overexpressing proNGF on activating RhoA kinase *in vivo* and *in vitro*. As shown in Figure 5B and 5C, proNGF induced 1.7- and 1.6-fold increase in active RhoA *in vivo* and in RGC-5 cells, respectively as compared with the control groups. Recent findings demonstrated proinflammatory effects of proNGF/p75^NTR^ via stimulating TNF-α expression, which can induce RGC death [29], [30]. As shown in Figure 5E, overexpression of proNGF in healthy retina induced TNF-α mRNA expression (3-fold) as compared with the control group. This effect was partially and significantly reduced (1.9-fold) by treatment with Y27632. We next compared the direct effects of proNGF versus TNF-α on activating RhoA in retinal ganglion cells. Cultures of primary retinal ganglion cells or RGC-5 were stimulated with proNGF (50 ng/ml) or TNF-α (10 ng/ml). Mutant proNGF induced activation (1.6-fold) of RhoA in RGC-5 cells (Fig. 5D) as detected by pull down assay and activation (1.75-fold) of RhoA in primary RGC cultures (Fig. 5F) as detected by G-LISA. In contrast, TNF-α caused modest increase in RhoA activation (20%) in both RGC-5 (Fig. 5D) and primary cultures as compared with controls (Fig. 5F).These results were further confirmed with complete blockade of active RhoA in groups treated with the selective Rho kinase inhibitor Y27632 *in vivo* and *in vitro*.

The article "Diabetes and Overexpression of proNGF Cause Retinal Neurodegeneration via Activation of RhoA Pathway" was retracted in 2017. Reasons: an official misconduct investigation; misconduct by an author; duplicated images.

**Figure 5:** ProNGF selectively activates RhoA kinase activation in vivo and in RGC cultures. **A.** Pull-down assay of rat retinal lysate showed 2.3-fold increase in the expression of active Rho in diabetic rats as compared with the controls (n = 4–5). **B.** Pull-down assay of rat retinal lysate showed 1.7-fold increase in active RhoA expression in rats electroporated with proNGF as compared with those electroporated with GFP (n = 5). **C.** Pull-down assay of RGC-5 lysate showed 1.6-fold increase in RhoA expression in RGC-5 cells treated with proNGF as compared with the controls (n = 4). Treatment of rats or RGC-5 with Y27632 blocked RhoA activation proNGF-treated samples but not the control groups. **D.** Pull-down assay of RGC-5 showing that treatment of RGC-5 cells with TNF-α did not increase RhoA activation as compared with the control group (n = 4). **E.** Statistical analysis showing overexpression of proNGF in healthy retina induced 3-fold increase in TNF-α mRNA expression as compared with the control group. **F.** Statistical analysis of G-LISA showing 1.7-fold increase of RhoA in primary RGC cultures treated with proNGF as compared with the control. TNF-α caused modest increase in RhoA activation (20%) as compared with the controls. These effects were reduced by treatment with Y27632. * = significant difference as compared with the control group at p<0.05.

### Inhibiting RhoA kinase blocked proNGF-induced p38/JNK MAPK activation

We next evaluated the activation of p38/JNK MAPK as a common signaling pathway implicated in neuronal death [2]. WB analysis of rat retinal lysate showed 1.5- and 1.8-fold increase in the phosphorylation of p38MAPK and JNK, respectively in proNGF group compared with GFP group (Fig. 6A, 6B). Furthermore, WB analysis of RGC-5 lysate showed 2.4 and 1.9-fold increase in the phosphorylation of p38MAPK and JNK, respectively in RGC-5 cells treated with mutant proNGF compared with the control (Fig. 6C, 6D).

The article "Diabetes and Overexpression of proNGF Cause Retinal Neurodegeneration via Activation of RhoA Pathway" was retracted in 2017. Reasons: an official misconduct investigation; misconduct by an author; duplicated images.

**Figure 6:** Inhibiting Rho kinase blocked proNGF-induced p38/JNK MAPK activation. **A,B.** WB analysis of rat retinal lysate showed 1.6- and 1.8-fold increase in the phosphorylation of p38MAPK and JNK in rats electroporated with proNGF as compared with those electroporated with GFP (n = 4–6). **C,D.** WB analysis of RGC-5 lysate showed 2.4 and 1.9-fold increase in the phosphorylation of p38MAPK and JNK, respectively in RGC-5 cells treated with proNGF as compared with the controls (n = 4). Treatment of rats or RGC-5 with Y27632 blocked all these effects in rats and media treated with proNGF and did not affect the control groups. * = significant difference as compared with the rest of the groups at p<0.05. C, control.

### Inhibiting RhoA kinase blocked diabetes- and proNGF-induced apoptotic markers expression

The expression of apoptotic markers was examined *in vivo* and *in vitro*. As shown in Figure 7A, 7C, diabetic rat retinal lysate showed 1.7-fold and 2.3-fold in the expression of cleaved-PARP and caspase-3 as compared with the controls. In parallel, there was 1.9- and 2.2-fold increase in the expression of cleaved PARP and caspase-3 in proNGF group compared with GFP-control (Fig. 7B, 7D). Treatment of rats with Y27632 blocked these effects. In addition, treatment of RGC-5 cells with mutant proNGF caused 2.1- and 1.6-fold increase in the expression of cleaved PARP and caspase-3 as compared with the controls (Fig. 7E). Co-treatment of RGC-5 with Y27632 blocked these effects.

**Figure 7:** Inhibiting Rho kinase blocked diabetes- and proNGF-induced apoptotic markers expression. **A,C.** WB analysis showing 1.9- and 2.2-fold increase in the expression of cleaved PARP and caspase-3 in rats electroporated with proNGF as compared with the controls (n = 4–5). **B,D.** WB analysis showing 1.9- and 2.2-fold increase in the expression of cleaved PARP and caspase-3 in RGC-5 cells treated with proNGF as compared with the controls (n = 4). **E.** WB analysis showing 2.1- and 1.6-fold increase in the expression of cleaved PARP and caspase-3 in RGC-5 treated with proNGF as compared with the controls. Treatment of rats or RGC-5 with Y27632 blocked all these effects in rats and media treated with proNGF and did not affect the control groups. * = significant difference as compared with the rest of the groups at p<0.05. C, control.

## Discussion

The main findings of the current study are: 1) Overexpression of the proNGF mimics diabetes action resulting in retinal neurodegeneration *in vivo* and *in vitro*, 2) Inhibiting Rho kinase exerted neuroprotective effects by inhibiting p75^NTR^ expression, inhibiting inflammation and activation of JNK/p38MAPK in response to proNGF or diabetes (Fig. 8). We believe that this is the first study to demonstrate a direct apoptotic effect of proNGF on retinal ganglion cells and delineate the apoptotic role of RhoA activation in retinal neurodegeneration. Together, these results support inhibition of RhoA kinase as a potential effective therapeutic target for the treatment of diabetic retinopathy.

The article "Diabetes and Overexpression of proNGF Cause Retinal Neurodegeneration via Activation of RhoA Pathway" was retracted in 2017. Reasons: an official misconduct investigation; misconduct by an author; duplicated images.

**Figure 8:** Diagram depicting the proposed role of proNGF/p75^NTR^ in diabetic retinopathy. Retinal neurodegeneration is thought to be induced via direct activation of RhoA kinase in RGC and paracrine inflammatory action in response to increases in proNGF.

Diabetes and proNGF overexpression caused significant increases in number of TUNEL-positive cells (Fig. 1) and loss of total neuronal cells and RGC in the ganglion cell layer (Fig. 2). Interestingly, while loss of total neuronal cells in GCL was 20–30%, specific loss of RGC identified by Brn3a, the selective RGC marker was 60%, suggesting that RGC cells are more sensitive to death signals in response to proNGF. These results lend further support to previous reports showing retinal neurodegeneration in response to diabetes or proNGF overexpression [1], [7], [23], [29]. Although it has been documented that proNGF can promote neuronal apoptosis through binding p75^NTR^ (reviewed in [3], [4]), the exact molecular events by which proNGF mediates its apoptotic action in retinal neurons are not fully understood. Whether RGCs express p75^NTR^ remains a controversy. We and others have demonstrated p75^NTR^ expression in both Müller cells and RGCs [1], [31]–[34], while other groups have reported p75^NTR^ expression only in Müller cells [29], [35], [36]. Findings from the current study support a direct apoptotic effect of proNGF on RGC (Fig. 3) as well as demonstrates p75^NTR^ expression in primary RGC cultures isolated from neonatal retinas (Fig. 4F) and mixed neuronal cultures isolated from adult retina (Fig. 4G). One possible explanation of these seemingly contradictory findings is that p75^NTR^ expression in RGC varies depending on the health and age whether developing or adult retina.

Overexpression of p75^NTR^ constitutively activates endogenous RhoA [8], [9] leading to neuronal death. Therefore, we hypothesized that inhibition of Rho kinase is neuroprotective. In agreement, our results showed significant activation of RhoA in diabetic retina, proNGF overexpressing retina and RGC cultures using pull down assay (Fig. 5A–C). Due to sample limitation, activity of Rho GTPase was detected using G-LISA technique in primary RGC cultures. These results also showed that mutant proNGF markedly (1.75-fold) causes Rho GTPase activity (5.E). Therefore, we examined the neuroprotective effects of RhoA kinase inhibitor Y27632, the first identified specific inhibitor of the ROCK family of protein kinases, in diabetic retinas as well as in response to proNGF *in vivo* and *in vitro*. Treatment with Y27632 showed significant neuroprotective effects both in diabetic animals (Fig. 1) and proNGF overexpressing retina (Figs. 1 and 2). *In vitro*, Y27632 completely blocked proNGF-induced cell death in primary RGC cultures and RGC-5 cell line. Of note, primary RGC cultures were far more sensitive to the apoptotic effects of proNGF compared to RGC-5 cell line (Fig. 3). Our results lend further support to previous reports showing neuroprotective of Y27632 in cultured cortical neuronal cells [37] and in models of cerebral ischemia and transient retinal ischemia [38], [39]. Although inhibitors of both Rho kinase and Rho GTPase have been shown to enhance ocular blood flow, retinal ganglion cell survival (reviewed in [40]), we believe that this is the first study to document the neuroprotective effects of Y27632 in diabetic retina or proNGF overexpression models.

The article "Diabetes and Overexpression of proNGF Cause Retinal Neurodegeneration via Activation of RhoA Pathway" was retracted in 2017. Reasons: an official misconduct investigation; misconduct by an author; duplicated images.

In addition to the direct apoptotic effect of proNGF/p75^NTR^ in neurons, a proinflammatory role of proNGF/p75^NTR^ has been proposed in Müller glial cells. We and others have shown that proNGF overexpression can induce marked retinal neuronal death via p75^NTR^-mediated TNF-α production in Müller glia cells [29], [30]. Inhibition or genetic deletion of p75^NTR^ exerted neuroprotective effects [29], [30], [41]. To investigate the effects of inhibiting Rho kinase activity on proNGF proinflammatory effects, we assessed TNF-α expression using rtPCR. The results showed that proNGF induced 3-fold increase in TNF-α expression that was partially but significantly reduced by Y27632 (Fig. 5E). These results support a proinflammatory role of proNGF in the retina and indicate that the neuroprotective effects of inhibiting RhoA could be attributed, at least in part to inhibiting inflammatory mediators including TNF-α. Accordingly, previous reports have shown that Y-27632 inhibited production of TNF-α via modulation of NFκB in non-diabetic models [42], [43]. Interestingly, our analyses showed that proNGF could activate RhoA in primary RGC cultures (1.75-fold) and RGC-5 cell line (1.6-fold) while TNF-α caused modest activation (20%) in both primary RGC and cell line (Fig. 5).These results support the direct and unique pathway proposed for proNGF activating RhoA apoptotic signal in RGC.

Activation of p38 and JNK in sensory neurons has been reported in early diabetes in rats and in diabetic patients [44]. In parallel, studies have also shown that activation of the RhoA/p38 MAPK pathway causes neuronal death [8]–[12]. In agreement, our results showed significant increases in phosphorylation of JNK and p38 MAPK in response to overexpression of proNGF in rat retina or RGC-5 cells. Treatment of the diabetic animals, proNGF-overexpressing animals or RGC-5 cultures with Y27632 prevented neuronal cell death and blocked expression of apoptotic markers including cleaved PARP. These results demonstrate a novel pathway by which increased expression of proNGF leads to retinal neurodegeneration directly via activation of p75^NTR^/RhoA in RGC. Inhibition of Rho/ROCKs might be an attractive therapeutic target in the treatment of diabetic retinopathy; however further studies are warranted to determine the role of ROCK inhibitors in clinical practice [45].
